# CMV-Independent Lysis of Glioblastoma by *Ex Vivo* Expanded/Activated Vδ1+ γδ T Cells

**DOI:** 10.1371/journal.pone.0068729

**Published:** 2013-08-07

**Authors:** Andrea Knight, Hilal Arnouk, William Britt, G. Yancey Gillespie, Gretchen A. Cloud, Lualhati Harkins, Yun Su, Mark W. Lowdell, Lawrence S. Lamb

**Affiliations:** 1 The Department of Haematology, University College London, London, United Kingdom; 2 Department of Medicine, University of Alabama at Birmingham School of Medicine, Birmingham, Alabama, United States of America; 3 Department of Pediatrics, University of Alabama at Birmingham School of Medicine, Birmingham, Alabama, United States of America; 4 Department of Surgery, University of Alabama at Birmingham School of Medicine, Birmingham, Alabama, United States of America; The University of Chicago, United States of America

## Abstract

Vδ2^neg^ γδ T cells, of which Vδ1+ γδ T cells are by far the largest subset, are important effectors against CMV infection. Malignant gliomas often contain CMV genetic material and proteins, and evidence exists that CMV infection may be associated with initiation and/or progression of glioblastoma multiforme (GBM). We sought to determine if Vδ1+ γδ T cells were cytotoxic to GBM and the extent to which their cytotoxicity was CMV dependent. We examined the cytotoxic effect of *ex vivo* expanded/activated Vδ1+ γδ T cells from healthy CMV seropositive and CMV seronegative donors on unmanipulated and CMV-infected established GBM cell lines and cell lines developed from short- term culture of primary tumors. Expanded/activated Vδ1+ T cells killed CMV-negative U251, U87, and U373 GBM cell lines and two primary tumor explants regardless of the serologic status of the donor. Experimental CMV infection did not increase Vδ1+ T cell - mediated cytotoxicity and in some cases the cell lines were more resistant to lysis when infected with CMV. Flow cytometry analysis of CMV-infected cell lines revealed down-regulation of the NKG2D ligands ULBP-2, and ULBP-3 as well as MICA/B in CMV-infected cells. These studies show that *ex vivo* expanded/activated Vδ1+ γδ T cells readily recognize and kill established GBM cell lines and primary tumor-derived GBM cells regardless of whether CMV infection is present, however, CMV may enhance the resistance GBM cell lines to innate recognition possibly contributing to the poor immunogenicity of GBM.

## Introduction

High-grade gliomas such as glioblastoma multiforme (GBM) can initiate and progress to an unsalvageable point without generating a significant immune response, consistent with Medawar's description of the brain as a site of relative immune protection [1]. Human cytomegalovirus (HCMV) infection has also been detected in a large percentage of human high-grade gliomas, and recent studies suggest a relationship between HCMV infection and initiation and/or progression of GBM [2]–[6]. The presence of latent CMV infection in GBM could present an opportunity for CMV-based immunotherapy, provided that such an approach could overcome the highly immunosuppressive microenvironment [7]–[11].

T cells bearing the γ and δ receptor (γδ T cells) are important effectors against malignancy-associated viral infections such as EBV [12] and HSV [13]. Indeed, increases principally in circulating Vδ1+, and to a lesser extent Vδ3+ and Vδ5+ T cell subsets [14], have been strongly and positively correlated with a response to and subsequent resolution of HCMV viremia [15]. Most importantly, CMV-reactive Vδ1+ γδ T cells also are cross-reactive against several malignant cell lines [15]–[18].

The Vδ1 subset is normally <10% of circulating γδ T cells but predominant in epithelial tissues. Vδ1+ T cells are activated by stress-induced self-antigens such as MIC-A/B and UL-16 binding proteins through the T cell receptor and NKG2D [19]–[21] and recognize glycolipids presented by CD1c on the surface of immature dendritic cells and can induce DC to mature and produce IL-12 [22], [23]. This population comprises cells that are highly cytotoxic to a wide variety of malignancies [24]–[29], and long-term persistence of Vδ1+ T cells in bone marrow transplant patients has been associated with long-term disease free survival [30], [31]. Vδ1-expressing T cells can also exhibit immunosuppressive and regulatory properties in addition to effector function [32], [33], a finding of particular importance in determining the interaction of γδ T cells and malignancy. We have previously shown that *ex vivo* expanded/activated γδ T cells are highly cytotoxic to glioma cell lines and primary GBM cell line explants, and that these γδ T cells will slow tumor progression and increase survival in immunodeficient mice bearing GBM cell line xenograft tumors [34], [35]. Separately, we also showed that γδ T cells are globally reduced in GBM patients although the proportion of circulating Vδ1 T cells was increased [36]. In this report, we build on previous work detailed above to determine if a Vδ1+ T cell response is evident in GBM patients, the potential for Vδ1+ T cell-mediated immune reactivity against GBM, and the extent to which CMV infection in high-grade gliomas affects their immunogenicity to Vδ1+ T cells.

## Materials and Methods

### Patients and healthy volunteers

Patients presenting with CT or MRI evidence of probable GBM were accrued for this study and enrolled following histological diagnosis. Patients and controls were excluded if they had been diagnosed with a co-existing immune system disorder; active viral, bacterial or parasitic infection; or prior organ or bone marrow transplant. The University of Alabama at Birmingham (UAB) Institutional Review Board for Human Research approved this study. Written informed consent was obtained from each patient or a designated family member. Written informed consent was obtained from healthy volunteers following explanation of the research studies.

### Expansion of Peripheral Blood γδ T cells and tumor-infiltrating lymphocytes

Two methods were used to expand peripheral blood γδ T cells from healthy volunteers and GBM patients (*n* = 5/group), one that preferentially expands the Vγ9Vδ2 cell population (ZOL/IL-2) and another that inhibits apoptosis in all γδ T cell subsets (CD2/OKT-3). In the ZOL/IL-2 method, mononuclear cells (MNC) were obtained by density gradient centrifugation and resuspended at 1.0×10^6^/ml in RPMI 1640+10% autologous serum +1 µM Zoledronate (Novartis Oncology; East Hanover, NJ) +50 U/ml IL-2 (Roche: Indianapolis, IN). The culture was maintained at the original density for 14d with addition of 50 U/ml IL-2 on post-culture days 2, 6, and 10 and addition of complete media as determined by pH and cell density. In the CD2/OKT-3 method described by Lopez [37], cultures were initiated in RPMI-1640 supplemented with L-glutamine, and 10% human serum 10% 1 M HEPES, 1,000 U/ml human rIFN-γ, 10 U/ml human rIL-12, and 1 µg/ml mouse anti-human CD2 mAb clone CLB-CD2 6G4 (Baxter Oncology, Deerfield, IL). Twenty-four hours later, 10 ng/ml anti-CD3 mAb OKT3 (Ortho Biotech) and 300 U/ml recombinant-human (rHu) IL-2 were added to the culture media and maintained at the original density for 14 d with addition of complete media as determined by pH and cell density. Tumor-infiltrating lymphocytes cultures were initiated from fresh GBM tumors from operative specimens. Tissues were minced finely with #11 scalpel blades followed trypsin and collagenase type IV for 2 h at room temperature. After digestion, the cells were washed twice in RPMI1640 and cultured using only the CD2/OKT-3 method as described above and maintained for 14 d with the addition of fresh complete media as needed.

### Expansion and activation of Vδ1+ γδ T cells from healthy volunteers

Up to 50 ml of peripheral blood was obtained from healthy volunteers. Peripheral blood mononuclear cells (PBMC) were isolated by density gradient centrifugation and resuspended at a concentration of 1×10^6^ cells/ml in RPMI-1640 supplemented with 10% pooled human serum. Vδ1+ T cells were sorted from PBMC using anti-Vδ1 (R9.12 Beckman Coulter) and ferromagnetic particles (Miltenyi Biotech; Bergen Gladbach, Germany). Purified Vδ1 T cells were expanded in 200 IU/ml recombinant IL-2 (R&D Systems; Abingdon, UK), 1 µg/ml PHA-L (Sigma-Aldrich; Taufkirchen, GE) and irradiated allogeneic PBMC feeder cells. After 3 weeks of culture, the resulting effector lines were phenotyped and purity (routinely >95%) was determined by multicolor fluorescent staining.

### Cell Lines

U251, U87, and U373 are established GBM cell lines that were obtained from the Brain Tumor Tissue Facility at UAB and have been verified to be authentic by short-tandem repeat PCR conducted by the UAB Cancer Genomics Core Facility (Michael Crowley, Director). The U87 is a grade IV glioma that originated from a 44-year-old Caucasian woman [38]. The genetic characteristics of the cell line have been well described [39]. The UAB Brain Tumor Tissue Core, a unit of the UAB NCI SPORE in Brain Cancer, obtained the cell line from the ATCC. Its origin has been verified by STR PCR and has been found to agree with the original cell source. U251MG is a grade III astrocytoma that was cultured from a 61 year old male [38] and was obtained directly from Darell D. Bigner (Duke University) who obtained them from Jan Ponten of Uppsala University. The cell line has been verified as authentic (Rb-deleted, p15/p16 wild type) and has the same STR pattern as the original line. U373MG has been previously identified as a subclone of the U251 cell line [40]. Cell lines were cultured in a 50∶50 mixture of Dulbecco's Minimum Eagle's Medium and Ham's Nutrient Mixture F-12 (DMEM/F12 50∶50) enriched with 7% heat inactivated pooled human cGMP-grade serum (Labquip; Woodbridge, ON), 2 mM L-glutamine and 10% Penicillin-Streptomycin-Amphotericin (Mediatech; Herndon VA). The human fetal lung fibroblast line MRC5 was obtained from European Collection of Cell Cultures (ECACC). Cells were cultured in MEM supplemented with 2 mM L-glutamine, nonessential amino acids (all from Sigma Aldrich) and 10% FCS. Fibroblasts were used between 32–40 passages and were maintained at 37°C in a humid atmosphere containing 5% CO2.

### Primary Tumor Explant Cultures

Short-passage primary GBM cultures were initiated from intraoperative specimens obtained from accrued patients. Tissue for explant was transferred aseptically into T75 flasks in about 15 ml of “complete culture medium” which is DMEM/F12 50∶50 (Mediatech; Herndon VA) supplemented to 7% with heat-inactivated fetal bovine serum and 2.6 mM L-glutamine. The medium was exchanged after 5–7 days and any cells growing out from the explants were maintained in primary culture. The cultures were monitored for growth and confluence and the media was changed weekly. Once cells on the flask were confluent, the cells were detached using trypsin and passaged and/or cryopreserved.

### Immunohistochemistry

Paraffin embedded sections of primary GBM were used for immunohistochemistry. Antibodies and sources were as follows: HCMV IE-1 (Millipore: Billerica, MA), MIC A/B (Bio Legend; San Diego, CA), ULBP-1, ULBP-2, ULBP-3, and ULBP-4 (Santa Cruz Biotechnology; Santa Cruz, CA). Sections of normal brain served as the antibody control and sections not labeled with primary antibody served as control for background. Specimens were deparaffinized in xylene and rehydrated by ethanol washes at decreasing concentrations (100%, 95%, 70%) followed by PBS. Boiling the sections for 5 min with EDTA in the pressure cooker was performed for antigen retrieval. Endogenous peroxidase quenching was performed with 3% peroxide for 5 min and rinsed with Tris buffer. 3% normal goat serum was then applied as a blocking agent for 20 min. Primary antibody was applied for one hour. Goat anti-mouse/anti-rabbit secondary antibody (Biogenex, San Ramon CA) was applied for 20 minutes followed by HRP for 20 min. Diaminobenzidine tetrahydrochloride (DAB) (Biogenex, San Ramon CA) was then applied for ∼8 min. After DAB staining, slides were rinsed with DI water and counterstained with pure hematoxylin for 45 s. Then the slides were dehydrated with graded ethanol and xylene and mounted in coverslips.

### *In situ* hybridization

For detection of HCMV nucleic acids, a biotinylated 21-base oligonucleotide (5′-GTGGTGGCGCTGGGGGTGGCG-3′) specific for HCMV early gene mRNA and biotinylated positive (specific for polyadenylic mRNA) and negative control (specific for HSV-1/2) probes were obtained (Novocastra; Buffalo Grove, IL). We performed enzyme digestion and nucleic acid denaturation of paraffin sections using a Misha thermocycler (Shandon Lipshaw, Pittsburgh, PA), and slides were hybridized overnight at 37°C in a humidified chamber (methods are detailed in manuscript in preparation). 4 Probe was detected using a supersensitive detection system (BioGenex, chromogen NBT). To detect HCMV DNA, we used a digoxigenin-labeled HCMV total genome DNA probe (Zymed Labs, South San Francisco, CA). The manufacturer provided positive (specific for endogenous alu DNA sequence) and negative (nonspecific DNA) digoxigenin-labeled control probes.

### CMV strains, infection procedure

Both clinical CMV strains TB40/E and VHL/E were kindly provided by Dr. Christian Sinzger (University of Tubingen, Germany). For infection, 5×10^5^ MRC5 fibroblasts per well were seeded into 24-well plate 24 h before adding the virus. Sub-confluent monolayers of MRC5 fibroblasts were incubated with CMV in suspension at multiplicity of infection (MOI) of 1–5 for 2 h at 37°C. After virus adsorption, cells were washed and cultured for 2–4 days. Infection was verified by microscopy to determine the cytopathic effect.

### Cytotoxicity assays

Targets are labeled with the membrane dye PKH26 (Sigma; St. Louis, MO). Expanded/activated γδ T cells are then added to the tubes at ratios of 0∶1 (Background), 5∶1, 10∶1, 20∶1 and 40∶1 effectors/GBM targets, incubated for four hours at 37°C and 5% CO_2_, washed ×1 and resuspended in 1 ml HBSS. To-Pro Iodide solution (Molecular Probes; Eugene, OR) 20 µl is added prior to acquisition on the flow cytometer. Cytotoxicity is calculated by dividing the number of PKH26+ToPro Iodide+ events by the total number pf PKH16+ events and multiplying the result by 100.

### Statistical methods

Descriptive statistics and nonparametric analysis using the Wilcoxon log-rank test was used to test for differences in expansion of γδ T cells observed between healthy donors and GBM patients and differences cytotoxicity of Vδ1+ T cells between CMV+ and CMV− donors. Where applicable, paired-ttests were used to compare cytotoxicity data and NKG2DL expression (data normally distributed).

## Results

### Peripheral blood γδ T cells obtained from patients prior to treatment and GBM-infiltrating γδ T cells obtained from resected tumor show minimal response to *ex vivo* stimulation

We previously reported that the proportion of circulating Vδ1+ T cells is increased in GBM patients and that the absolute Vδ1+ T cell count did not significantly differ from older healthy volunteers [36]. In these experiments, we cultured peripheral blood mononuclear cells (MNC) from five GBM patients in an effort to determine whether the Vδ1+ T cells could respond to *ex vivo* stimuli and whether sufficient numbers of cells could be obtained for cloning and assay for anti-CMV activity. As shown in ***Figure 1***, γδ T cells from patients with GBM failed to expand using either the ZOL/IL-2 or CD2/OKT-3 culture conditions. Less than 5-fold expansion was seen in all peripheral blood specimens from GBM patients by both methods, neither of which showed a significant advantage in expanding γδ T cells from GBM patients (p = 0.12). In contrast, γδ T cells from healthy volunteers expanded well using CD2/OKT-3 (n = 7, median = 200 with range 100 to 375 fold) or ZOL/IL-2 (n = 5, median = 223 fold, range 46 to 435 fold). Few γδ T cells were seen in tumor infiltrating lymphocytes (TIL) preparations obtained from freshly resected GBM tumors and these also did not respond to T cell stimulation culture. *(* ***Figure 2*** *)*.

**Figure 1:** Flow cytometry dot plots γδ T cell expansion cultures of peripheral blood from five pre-resection GBM patients and one healthy volunteer. The γδ T cells were expanded/activated by either *(a)* CD2/OKT-3 or *(b)* ZOL/IL-2 methods as described in the text. Peripheral blood from a representative healthy control is shown at right. After 14 days in culture, neither method was effective in expanding γδ T cells from the blood of any of the five GBM patients although γδ T cells from healthy volunteers were readily induced to proliferate (p = 0.12 for both methods).

**Figure 2:** Culture of tumor infiltrating lymphocytes (TIL) from a representative human GBM. Note an initial very low percentage of γδ T cells that could not be expanded in two week culture using the CD2/OKT3 method (see text). Flow cytometric dot plots were gated on CD3+ lymphocytes. Similar results were obtained from three additional patients.

### Cultured Vδ1+ T cells from CMV-seronegative and CMV-seropositive healthy volunteers lyse standardized glioma cell lines and short-passage primary explants from GBM tumors equally well

Vδ1+ T cells from CMV- (Donor 1) and CMV+ (Donor 2) healthy volunteers cultured using a standardized culture method developed in our laboratory [18] consistently yielded over 90% Vδ1+ T cells *(* ***Figure 3a*** *)* and efficiently lysed glioma cell lines U87, U251 and U373 and primary GBM explants designated 1016 and 1042 *(* ***Figure 3b*** ***and Figure s1*** *)*. Expanded/activated Vδ1+ T cells were not cytotoxic to cultured human astrocytes in E∶T ratios up to 20∶1. Cytotoxicity against CMV-infected astrocytes was <5% at the highest E∶T ratio (20∶1) assessed. Additional experiments that incorporated cytolytic activity of Vδ1+ T cell cultures from CMV seropositive (n = 4) and CMV seronegative (n = 6) donors against U251 cells and the GBM primary explant line 1042 *(* ***Figure 3c*** *)* revealed no significant impact on cytotoxicity based on CMV serologic status (p = 0.75 and p = 0.29 respectively).

**Figure 3:** Cytotoxicity of expanded/activated Vδ1+ T cells from CMV seropositive and seronegative healthy volunteers against human glioma cell lines. (***a***) Flow cytometric analysis of 14-day expansion culture of purified Vδ1+ T cells from two healthy volunteer donors. (***b***) Cytotoxicity of purified and expanded Vδ1+ T cells from two donors against three (left to right for each donor) GBM cell lines (*a*) U251, (*b*) U87, and (*c*) U373 and two primary cell lines from GBM explants designated (d)1016 and (*e*)1042 in a four-hour cytotoxicity assay at an E∶T ratio of 20∶1. (***c***) Vδ1+ T cell cultures were expanded from additional CMV-seropositive (n = 4) and CMV-seronegative (n = 6) donors as described in the text and reacted over 4 h at an E∶T ratio of 20∶1 is shown with the U251MG glioma cell line and the 1024 primary GBM explant line. Donor CMV serologic status had no effect on Vδ1+ T cell cytotoxicity against U251 (p = 0.75) or 1042 (p = 0.29), respectively for CMV seropositive and CMV seronegative donors.

After establishing that Vδ1+ T cells are cytotoxic to GBM cells, we next considered whether this Vδ1+ T cell-mediated recognition and lysis of primary glioma explants could be associated with latent CMV infection. Indeed, the two primary GBM tumors from which cell explants 1016 and 1042 were derived expressed CMV-associated antigens IE-1 and pp65 *(* ***Figure 4a*** *)* as well as CMV mRNA *(* ***Figure 4b*** ***, upper panel*** *)*. CMV mRNA was also detectable in both cell lines *(* ***Figure 4b*** *)* suggesting continued CMV infection. As expected and previously reported, there was no evidence of deep parenchymal T cell invasion of these tumors *(* ***Figure 4a*** *)*. Strong expression of Vδ1+ T cell target NKG2D ligands (NKG2DL) ULBP-2 and ULBP-3 and moderate expression of ULBP-1 was noted on both tumor cell lines. There was little to no expression of MIC-A/B on either line *(* ***Figure 5*** *)*.

**Figure 4:** Assessment of CMV activity in primary GBM and derived cell lines. (a) Primary GBM from which cell explants 1016 and 1042 were derived expressed CMV-associated surface antigens IE-1 and pp65, although T cell invasion beyond perivascular areas as indicated by anti-CD3 labeling is minimal. (b) Both primary tumors 1016 and 1042 (top panel) were assessed for the presence of CMV mRNA by in-situ hybridization using a biotinylated 21-base oligonucleotide (5′-GTGGTGGCGCTGGGGGTGGCG-3′) specific for HCMV early gene mRNA and a biotinylated positive (specific for polyadenylic mRNA) and negative control (specific for HSV-1/2) probe. provided positive (specific for endogenous alu DNA sequence) and negative (nonspecific DNA) digoxigenin-labeled control probes. Both tumors show the presence of CMV mRNA as do the short passage cell lines that were derived from them (bottom panel) suggesting continued CMV infection.

**Figure 5:** Assessment of stress antigen expression cell lines derived from primary GBM. Primary GBM cell line explants 1016 and 1042 were labeled with fluorochrome-tagged antibodies to respective isotype control anti-IgG (clear) and Vδ1+ T cell target NKG2DL MIC A/B, ULBP-1, ULBP-2 and ULBP-3 (shaded). Strong expression of ULBP-2 and ULBP-3 is noted. Primary 1042 is a heterogeneous tumor with a brightly autofluorescent subpopulation seen as a bimodal peak for both isotype and labeled plots.

### Experimental acute CMV infection of selected glioma cell lines is associated with a reduction of NKG2DL expression and in some cases reduced cytotoxicity

In order to determine the impact of CMV infection on tumor vulnerability to Vδ1+ T cells, we infected the CMV-negative glioma cell line U251 with CMV strain TB40/E and assessed Vδ1+ T cell cytotoxicity against both the infected and unmanipulated cell lines. Expanded/activated Vδ1+ T cells lysed both CMV-infected and unmanipulated U251 cells, although a significant reduction in cytotoxicity to CMV-infected U251 cells was noted at the E∶T ratio of 20∶1 (n = 6, p = 0.021). ***Figure 6a*** shows results of cytotoxicity assays against U251 from three representative donors. When examined separately, donor CMV serologic status (n = 3 seropositive and 3 seronegative) was not a factor in lysis of either infected or unmanipulated cells (p = 1.00 at 1∶20 effector∶target ratio, data not shown). ***Figure 6b*** compares NKG2DL expression between unmanipulated U251 cells and U251 cells that had been infected in culture for 5 days. MIC A/B and ULBP-2 were consistently down regulated in CMV-infected U251 cell cultures. ULBP-1 and ULBP-3 expression was variable between cultures. When CMV-infected U251 cells were assessed based on expression of HCMV-IE-1 expression *(* ***Figure 6c*** *)*, however, it was noted that cells strongly expressing IE-1 (red histograms) generally showed little change in MIC-A/B expression when compared to a parallel unmanipulated culture (black histograms). Unmanipulated cells do not express IE-1 (data not shown) and expressed all UL-16 binding proteins at higher density than CMV-infected cells. Interestingly, the IE-1^neg^ population (blue) showed only ULBP-2 expression. This population contains a mixture of fragile infected and non-viable cells many of which have shed these surface markers. Taken together, as Vδ1+ T cells are known to recognize NKG2D ligands as a mechanism for cytotoxic activity, these findings suggest that the extent to which different glioma cell lines regulate NKG2DL expression in response to CMV infection is variable and may be associated with partial protection from Vδ1+ T cell – mediated lysis.

**Figure 6:** CMV infection modulated NKG2DL expression on glioma cell lines and their vulnerability to lysis by Vδ1+ T cells. (a) Lysis of unmanipulated U251MG cells (filled circles) versus CMV-infected U251MG cells (open circles) by expanded/activated Vδ1+ T cells for three representative donors in a 4 h flow cytometric cytotoxicity assay. CMV-infected cells are more resistant to lysis (p = 0.021) at E∶T ratio of 20∶1. (b) Expression of NKG2DL on three cultures of unmanipulated (CMV-) vs. CMV-infected (CMV+) U251 glioma cultures as determined by Median Fluorescence Intensity (MFI) following acquisition of a minimum of 10,000 events. (c) Expression of NKG2DL on unmanipulated (black), HCMV IE-1 expressing (red) and IE-1^neg^ (blue) U251 glioma cells after 5 days of culture (see text).

## Discussion

In previous work we have shown that γδ T cell cultures cultured *ex vivo* using a combination of anti-CD2, OKT-3, and IL-2 are cytotoxic to high-grade gliomas *in vitro* and to human xenograft tumors in immunodeficient mice [34], [35]. We now extend our previous findings to examine the specific function of the Vδ1+ T cell population in the context of the immune response and potential immunotherapies for malignant glioma. Clinical data and murine models both support a vigorous γδ T cell response to CMV infection [14], [41] that is skewed toward Vδ2- in humans. This Vδ2- population is comprised principally of Vδ1+ T cells, a population with both cytotoxic and regulatory/suppressive roles in malignancy and infection [33]. Understanding of the function of Vδ1+ T cells in the immune response to cancer is currently limited, particularly with respect to glioblastoma tumors that have shown persistent CMV infection.

Strategies for expansion of circulating Vγ9Vδ2+ T cells have been elusive. Indeed, our laboratory and others have extensively reported poor persistence, death, and functional anergy of *ex vivo* expanded/activated Vγ9Vδ2+ T cells, particularly when they are obtained from cancer patients [35], [42]–[44]. *Ex vivo* expansion of Vδ1+ γδ T cells, however, has met with some success, particularly when cells are obtained from patients with neuroblastoma and myeloma [26], [45], [46]. Vδ1+ γδ T cells GBM patients, however, were resistant to *ex vivo* stimulation methods that readily expand this population in healthy volunteers and appear to be functionally anergic.

We then tested the cytotoxicity of *ex vivo* expanded Vδ1+ T cells from healthy volunteers against standardized glioma cell lines and two cultured explants derived from primary brain tumors grown in short-term culture to determine if CMV infection was associated with vulnerability to recognition and lysis. The two primary tumor explants designated 1042 and 1016 were effectively lysed by *ex vivo* expanded Vδ1+ T cells *(* ***Figure 3*** ***and Figure s1*** *)* and were shown to be positive for CMV infection both in sections from the primary tumors and the short-passage cell lines derived from them. We were able to demonstrate strong expression of pp65 and IE-1 as well as the presence of CMV mRNA in the primary GBM tumors from which the cell preparations were obtained. Cultured cells from these tumors also showed evidence of continued CMV infection *(* ***Figure 4*** *)* and expressed several stress-associated NKG2D ligands *(* ***Figure 5*** *)*. However, Vδ1+ T cells also consistently lysed U251MG, U87MG, and U373 GBM cell lines, which do not express CMV-associated antigens nor do they harbor replicating CMV. These findings are consistent with earlier work from this laboratory that documents significant CMV-independent cytotoxicity of purified Vδ1 T cells against leukemia and myeloma cell lines and primary leukemia [30], [31], [46].

Cytotoxicity of γδ T cells against tumor cells and virus-infected cell lines is broadly based and is generally related to expression of stress-associated surface proteins [19], [47]. We have previously shown that γδ T cells with strong cytotoxicity to glioma cell lines do not kill normal human astrocytes in culture [48], and in this work we have also shown that CMV-infected astrocytes are also not killed by cytotoxic Vδ1+ T cells. Separately, we have also shown essentially negative cytotoxicity toward uninfected vs. strong cytotoxicity toward CMV-infected MRC fibroblasts [18]. Taken together, these data strongly suggest that Vδ1+ T cell recognition and cytotoxicity against gliomas is at least in part modulated by expression of stress-induced NKG2DL and independent of latent or persistent CMV infection.

Although our findings suggest that Vδ1+ T cells were not dependent on CMV infection in order to recognize and lyse gliomas, Vδ1+ T cells potentially could recognize glioma cells based on previous exposure to CMV. This “crossover” cytotoxicity was first shown by Halary [16], who found that that Vδ2^neg^ T cells (of which Vδ1+ T cells are the predominant population) both recognize and respond to CMV-infected fibroblasts and lyse the HT-29 intestinal tumor cell line independent of CMV infection. Based on this previous work, we examined the cytotoxic function of expanded Vδ1+ T cells obtained from healthy CMV seropositive and seronegative donors against standardized glioma cell lines and against cells cultured from freshly resected GBM. We were unable to demonstrate any difference in cytotoxicity between Vδ1+ T cells expanded from either CMV+ or CMV− donors against the glioma targets *(* ***Figure 3*** *)*. These findings are consistent with earlier work that found that although an expanded and clonally restricted Vδ1+ T cell population could be documented both in CMV-seropositive and CMV- seronegative healthy individuals, the cytolytic response to CMV-infected fibroblasts was no different between the donor groups [18].

Having established that Vδ1+ T cell-mediated recognition and lysis was not dependent on CMV infection, we then asked whether CMV infection could potentiate or inhibit Vδ1+ T cell recognition of gliomas. When standardized CMV- glioma cell lines were artificially infected with CMV, Vδ1+ T cell cytotoxicity against glioma cell line targets was either less or the same at comparable effector∶target ratios *(* ***Figure 6*** *)*. CMV infection did not result in increased vulnerability of GBM cell lines to Vδ1+ T cell mediated cytotoxicity. Inhibition of Vδ1+ T cell cytotoxicity to CMV-infected GBM could occur through several mechanisms. Paradoxically, down-regulation of NKG2D has been shown in NK cells when exposed to CMV infected glioma, a response thought to be associated with control of the immune response to virus CMV infection [49], as has the sequestration of NKG2DL on infected cells [50]. Blocking of MIC-A/B and individual UL-16 binding proteins decreases cytotoxicity of γδ T cells to U251MG cells but do not abrogate cytotoxicity entirely [48]. Blocking of 4 NKG2DL simultaneously decreases cytotoxicity by approximately 40%, consistent with the reduced cytotoxicity seen in CMV-infected U251MG. Indeed, our findings detailed in ***Figure 6b*** shows modulation of MIC-A/B and ULBP-2 consistent with previous reports of UL-16 sequestration or modulation of expression in multiple NKG2D ligands in CMV-infected cells. [51], [52]. Taken together, these findings suggest that sequestration of NKG2DL MIC-A and ULBP-2 in CMV-infected U251MG cells is a contributing factor to decreased immunogenicity of glioma cells to recognition by NK and γδ T cells. These findings, however, must be interpreted in the context of experimental CMV infection, which is substantially different than the long-term latent CMV infection of GBM *in situ*. A further complication is the use of CMV strains that are propagated in the laboratory that may have critical differences from the CMV strains that have been isolated from GBM. Investigators have recently published an *in vitro* model of long-term CMV infection in a GBM cell line that can retain the virus in multiple passages which if reproducible and successful in animal models may reflect CMV interaction with GBM and the immune microenvironment with greater accuracy [53]

In summary, we have shown that pure cultures of expanded and activated allogeneic Vδ1+ γδ T cells are cytotoxic to primary glioma and glioma cell lines. Experimental CMV infection does not render the glioma cell lines more vulnerable to lysis by γδ T cells and in some cases will decrease immunogenicity by down-regulation of NKG2D ligands expression. In addition, γδ T cells from CMV-seropositive individuals do not show enhanced cross-reactivity to primary tumor explants or glioma cell lines as has been seen in other tumor types. These findings suggest that Vδ1+ γδ T cells are potent effectors against glioma, are not dependent of CMV infection for their cytotoxicity, and should be further explored in the design of immunotherapeutic strategies for high-grade brain tumors.

## Supporting Information

Figure S1 **Detail of Cytotoxicity of Vδ1+ T cells against glioma cell lines and primary GBM at a range of Effector∶Target ratios from** **Figure 3b** **.**
(TIF)
